# Effects of Different Particle Sizes of Hydroxyapatite on the Distribution and Migration of Trace Elements (Copper and Cadmium) in a Smelter-Impacted Soil

**DOI:** 10.1155/2021/2412646

**Published:** 2021-10-19

**Authors:** Lei Xu, Xiangyu Xing, Zhenqiu Zhu, Hongbiao Cui, Jianbiao Peng, Ding Li, Mingfei Ji, Jing Zhou

**Affiliations:** ^1^College of Environmental Science and Tourism, Nanyang Normal University, Nanyang 473061, China; ^2^Henan Key Laboratory of Ecological Security for Water Source Region of Mid-line of South-to-North Diversion Project, Nanyang 473061, China; ^3^College of Non-Major Foreign Language Teaching, Nanyang Normal University, Nanyang 473061, China; ^4^Key Laboratory of Soil Environment and Pollution Remediation, Institute of Soil Science, Chinese Academy of Science, Nanjing 210008, China; ^5^School of Earth and Environment, Anhui University of Science and Technology, Huainan 232001, China; ^6^School of Environment, Henan Normal University, Xinxiang 453007, China

## Abstract

To study the remediation effect of hydroxyapatite with different particle sizes, a field in situ experiment was carried out by adding conventional hydroxyapatite (0.25 mm) and microhydroxyapatite (3 *μ*m) and nanohydroxyapatite (40 nm) to the contaminated soil and planting *Elsholtzia splendens*. The distribution and migration of copper (Cu) and cadmium (Cd) in soil were investigated after 4 years. The results show that the application of three different particle sizes of hydroxyapatite significantly raise the soil pH, total phosphorus, and soil organic carbon. Moreover, the addition of hydroxyapatite can reduce the EXC fraction of Cu and Cd by 73.7%–80.1% and 20.8%–35.2%, respectively. In addition, the concentrations of Cu and Cd in >2 mm, 0.25–2 mm, 0.053–0.25 mm, and <0.053 mm aggregate are significantly increased. This improvement indicates that there are risks which may cause the increasing of total Cu and Cd in the soil where the pollution sources still exist. Furthermore, the content of soil colloid is significantly increased, and the colloidal Cu and Cd distribution percentage have been significantly increased by 49.9%–120% and 30.3%–181%. This result illustrates that the application of hydroxyapatite may greatly increase the possibility of colloid and dust migration of Cu and Cd.

## 1. Introduction

The contamination of heavy metals in soil has arisen much public concern both domestically and internationally [1, 2]. Previous studies have shown that activities such as mining and smelting can translocate heavy metals into the soil [3]. Meanwhile, excessive accumulation of heavy metals in soils not only reduces soil quality, microbial activity, and crop production but also threatens ecological security and human health [4]. During the past decades, more cost-effective and environmentally friendly techniques have been developed to reduce the harm of heavy metal contamination in soil on human and environment, including bioremediation and integrated remediation. Soil amendments have been widely used in in situ remediation of heavy metal contaminated soils due to their economic and in situ characteristics [5, 6].

A large number of studies have shown that phosphorus-containing materials (e.g., apatite, potassium dihydrogen phosphate, superphosphate, and hydroxyapatite) can effectively reduce the activities of heavy metals, such as Pb, Cd, and Cu in soil and wastewater [7]. Among them, hydroxyapatite has been widely used to remediate heavy metal contaminated soil and sediments owing to its strong adsorption and fixation ability for heavy metals [8, 9]. Although hydroxyapatite cannot reduce the total amount of heavy metal pollutants, it can be combined with heavy metals or transform them from active state to inactive state [10]. It has been demonstrated that the particle size of the material can significantly affect the bioavailability and geochemical stability of heavy metals in soil [11, 12]. However, the results about the influence of the particle size of hydroxyapatite on its passivation effect are controversial. Chen found that compared with phosphate rock powder with 35 *μ*m, the phosphate rock powder with 133–266 *μ*m can reduce the bioavailability of heavy metals in soil more effectively [13]. Dong's research results suggested that micro-nano hydroxyapatite whose particle size between microhydroxyapatite and nanohydroxyapatite was more helpful to reduce the availability of Cu and Cd in contaminated soil than microhydroxyapatite and nanohydroxyapatite [14]. In addition, researches on the immobilization of heavy metals in soil by hydroxyapatite are mostly completed in the laboratory, but there is a lack of comparative study on field restoration experiments [15]. More importantly, most of the studies about hydroxyapatite only focus on its effect on the heavy metal activity and bioavailability, but there are few researches paying attention to its potential effect on the distribution and migration of heavy metals in soil.

In this study, three different particle sizes of hydroxyapatite (conventional particle size, micro- and nanohydroxyapatite) were selected as test materials to study the existing forms, distribution, and migration of heavy metals in soil after 4 years of remediation in field scale. The objectives of this study were to (1) compare the effects of three particle size hydroxyapatite on the existing forms and chemical fractions of Cu and Cd in soil and (2) investigate the changes of Cu and Cd in the distribution and migration in the smelter-impacted soil. The results would put insight into the stabilization effect of different particle size materials in field scale and remind us to pay attention to the risk management and control of soil after remediation.

## 2. Materials and Methods

### 2.1. Study Site

The study site is located in Guixi City, Jiangxi Province, China (116°55′ E, 28°12′ N). The area has a subtropical monsoon climate, with an average annual precipitation of 1808 mm. Farmers had used water containing heavy metals to irrigate for a long time, which led to heavy metal contamination in soil (mainly Cu and Cd) and Cd concentrations in rice exceeding the national food health standards (GB 15201-94). The soil texture is sandy loam, and the pH is 4.63. The contents of soil organic carbon, total nitrogen, total phosphorus, total potassium, available nitrogen, available phosphorus, and available potassium are 16.3 g·kg^−1^, 1.33 g·kg^−1^, 0.261 g·kg^−1^, 2.38 g·kg^−1^, 67.1 mg·kg^−1^, 186 mg·kg^−1^, and 54.8 mg·kg^−1^, respectively. The concentrations of soil total copper and total cadmium are 517 mg·kg^−1^ and 0.410 mg·kg^−1^.

### 2.2. Reagent and Plants

Hydroxyapatite (pH = 8.40, particle size 0.25 mm) was purchased from Nanzhang Lihua mineral powder factory, Hubei, China; microhydroxyapatite and nanohydroxyapatite (pH = 7.68, particle size = 3 *μ*m; pH = 7. 72, particle size = 40 nm) were purchased from Emperor Nano Material Co. Ltd. (Nanjing, China). Cd and Cu concentration in hydroxyapatite, microhydroxyapatite, and nanohydroxyapatite were 1.18 mg·kg^−1^and 9.54 mg·kg^−1^, 3.83 × 10^−2^ mg·kg^−1^and 5.85 mg·kg^−1^, and 3.71 × 10^−2^ mg·kg^−1^ and 4.4 mg·kg^−1^, respectively. In our previous research, the transmission electron microscopy was used to analyze the morphology of these three different particle sizes of hydroxyapatite, and the transmission electron microscopy imaging of the different grain sizes of hydroxyapatite indicated that the shapes of HA, MHA, and NHA were bulk, spherical, and acicular, respectively (Figure 1) [16]. *Elsholtzia splendens*, which was a Cu-tolerant plant, was selected as the phytoextractor in this study.

### 2.3. Plot Design

The field experiments were conducted in triplicate and were designed with the land split into randomized plots. Each plot was 6 m^2^ (3 m × 2 m) and the plots were separated by plastic plates. The treatments applied were (1) 1% hydroxyapatite (HA) (w/w according to the mass of surface 17 cm soil, 22.3 t·ha^−1^, the same below), (2) 1% microhydroxyapatite (MHA), (3) 1% nanohydroxyapatite (NHA), and (4) the control (CK). The dosage chosen in the experiments was based on our previous experimental results [17]. The materials were applied in every plot on 26 December 2012. Then, they were mixed thoroughly with the soil by rotary tillage and then irrigated with tap water after the application of the materials (500 t·ha^−1^). *Elsholtzia splendens* were planted with a spacing of 30 cm × 30 cm (70 plants per plot) in every plot on April 26 in 2013, 2014, 2015, and 2016 with a compound fertilizer (N: P_2_O_5_: K_2_O = 15: 15: 15) before the plants were planted at a spreading of 0.833 t·ha^−1^. These hydroxyapatites were only applied at the start in 2012 during the study period 2012–2016.

### 2.4. Sample Collection

The test crop *Elsholtzia splendens* was harvested at the beginning of December every year. After the plant samples were harvested in 2016, five soil samples were collected from each plot in the 0–17 cm depth and fully mixed to form a composite soil sample (about 5 kilogram), the soil samples were divided into two portions: one portion was aired and ground in experiment for physicochemical and soil colloid analysis, and the other portion was aired for the aggregate analysis.

### 2.5. Sample Analysis

The soil pH was measured with a glass electrode at a water soil ratio of 2.5 : 1 (PHS-2CW-CN, Bante, Shanghai, China). Walkley–Black procedure was used to measure the soil organic carbon (SOC), total nitrogen (TN), and total phosphate (TP) [18]. Page's method was used to measure the soil available phosphate (HA) and nitrogen (AN) contents [19]. Soil total potassium (TK) and available potassium (AK) were measured according to Olsen [20]. The soil cation exchange capacity (CEC) was measured according to the ammonium acetate method [21].

The soil aggregates were divided into dry aggregate and wet aggregate and measured by the methods of Panettieri and Elliott [22, 23]. The dry aggregates were divided into aggregates sized >5 mm, 2–5 mm, 1-2 mm, 0.5–1 mm, 0.25–0.5 mm, and <0.25 mm, and the wet aggregates were divided into aggregates sized >2 mm, 0.25–2 mm, 0.053–0.25 mm, and <0.053 mm [24].

The Cu and Cd in whole soil, aggregates, and colloid were measured by atomic absorption spectrophotometry (SpectrAA-220) after the samples were digested [25]. The fractions of Cu and Cd were determined by the sequential extraction procedure [26]. In order to ensure the reliability of the experimental data, a standard soil sample (GBW07405, National Research Center for Certified Reference Materials, China) was used during the experiment. The percentage recoveries of heavy metals ranged from 96% to 107%.

The soil colloid was extracted by siphon method, and the settling time of soil colloid (<2 *μ*m) was calculated according to Stokes law [27]. After the soil colloid suspension was obtained, the content of soil colloid and heavy metal was determined by drying method. The settling time of soil colloid (<2 *μ*m) was calculated based on Stokes law. The contents of soil colloid and heavy metal in soil colloid were determined by drying method of Hu [28]. Briefly, 30 g of air-dried soil, which had passed the 2 mm pore size sieve, was added into 250 mL pure water, dispersing it with ultrasonic wave for 30 min. The dispersed suspension was washed into a 1000 mL high type beaker with 750 mL pure water. The soil colloids of less than 2 *μ*m were extracted by siphon method after stirring with glass rod for 1-2 min and settling for 6 h, 53 min, and 24 s. 20 mL soil colloid suspension was added into Teflon crucible by siphoning and dried at 50°C; then the content of soil colloid was determined by weighing method.

### 2.6. Statistical Analysis

SPSS20.0 (IBM SPSS, Somers, NY, USA) was used for one-way ANOVA and correlation analysis, and all the graphics were plotted by SigmaPlot 12.5.

## 3. Results and Discussion

### 3.1. Surface Soil Properties

The properties of surface soil in plots of the four treatments are summarized in Table 1, and there were no significant changes between different treatments in terms of the total N and K; however, the concentration of total P had been significantly increased by the application of HA, MHA, and NHA. This might be due to that as phosphorus-containing remediation materials, the application of three materials increased the content of total phosphorus in soil [25]. Meanwhile, the contents of available N, P, and K were significantly increased after the application of these three amendments. At the same time, the soil pH was greatly increased by 1.13–1.18 units after the application of HA, MHA, and NHA. Owing to hydroxyapatite being a kind of alkaline material which can consume a lot of H^+^ when dissolved [formula (1)], the presence of hydroxyapatite can decrease soil exchangeable acid and thus increase the soil pH [16]. The result was similar to a previous study, in which the addition of nanohydroxyapatite significantly increased soil pH by 1.8 units [29]. In addition, although the pH of HA is the highest, the results showed that the MHA had the best improvement on soil pH after three years remediation, followed by NHA and HA. This may be due to the fact that HA contains not only hydroxyapatite but also a certain amount of CaCO_3_, which can dissolve rapidly under acidic conditions, resulting in its less effective maintenance of soil pH than MHA and NHA [16]. The concentration of soil total nitrogen did not change significantly after remediation; however, the SOC contents in the 0–17 cm layer were significantly increased after the addition of HA, MHA, and NHA, and the highest content was found in the NHA (19.2 g·kg^−1^). This finding might be attributable to three reasons: (1) the vegetation restoration in this area increases vegetation coverage and reduces soil erosion and nutrient loss after the application of the three materials (Wang et al., 2018), (2) the presence of plant residues, roots, and root exudates also increased the input of organic matter to the soil [30], (3) the change in the microbial types and quantities is caused after cultivation that participated in soil organic matter degradation [31]. Thus, these changes could indirectly affect the content of the soil organic matter:

(1) $$\begin{array}{c} Ca_{10}{\left({\text{PO}}_{4}\right)}_{6}{\left(\text{OH}\right)}_{2}{+14\text{H}}^{+}{=10\text{Ca}}^{2+}{+\;6\text{H}}_{2}{\text{PO}}_{4^{-}}{+\;2\text{H}}_{2}\text{O} \end{array}$$

The total Cu content of soil did not significantly decrease after 3 years of remediation, while the concentration of total Cd in soil increased slightly. These results seemed to deviate from the goal of soil remediation, which was to reduce the concentration of heavy metals in soil, and similar results have been reported in our previous study in this region [25]. This might be due to the heavy metal pollution caused by dry and wet deposition in the air, although the area was no longer polluted by heavy metals brought by irrigation water. The research of Tao found that the contents of Cu and Cd in deposition in this area reached 1973 mg·m^−2^ and 15.2 mg·m^−2^, respectively [32]. In addition, by comparing heavy metal input (input of passivation material and atmospheric dry and wet deposition) and export (plant absorption, surface runoff and downward leaching), we found that the addition of passivation materials (conventional hydroxyapatite, lime, and charcoal) improved the adsorption and fixation capacity of Cu and Cd in soil, but the heavy metal output through surface runoff and leaching was reduced. As a result, the total Cd in the remediation surface soil was higher than that in the CK [33, 34]. Therefore, it is very important to completely cut off the input of foreign pollutants in the process of soil passivation remediation.

### 3.2. Chemical Fractions of Cd and Cu

Heavy metals in soil can be divided into solid and solution phases according to their existing forms, and they mainly exist in the solid phase [35]. Moreover, heavy metals in solid phase can be divided into different fractions according to their solubility, mobility, bioavailability, and potential environmental toxicity; therefore, a single extraction step cannot fully evaluate the toxicity and migration of heavy metals in soil [36]. In order to evaluate the migration and bioavailability of heavy metals in soil, a sequential extraction procedure was used in the present study. The different fractions of Cu and Cd in the soil are listed in Tables 2 and 3 , respectively. The distribution of five fractions of Cu was changed from RES > EXC > OM > Fe-Mn > CA to RES > Fe-Mn > OM > CA > EXC after the materials were applied. The application of the HA, MHA, and NHA could significantly decrease the EXC fraction of Cu (66.5%–80.1%) and increase the CA fraction and Fe-Mn fraction of Cu (94.1%–114% and 52.3%–71.5%). The application of the three materials had no significant effect on the OM fraction and RES fraction of Cu. This may be related to the mechanism of fixing heavy metals in soil by hydroxyapatite, which mainly reduces the activity of heavy metals through ion exchange, surface complexation, and coprecipitation [37, 38]. Similar to the chemical fraction of Cu, the application of materials significantly reduced the EXC fraction of Cd (20.8%–35.2%) and increased the Fe-Mn fraction of Cd (78.1%–127%). However, different from CA fraction of Cu, only MHA and NHA could significantly increase the CA fraction of Cd in soil (47.0% and 132%), and HA had no significant effect on the CA fraction of Cd.

The EXC fraction of Cu and Cd could be significantly reduced by MHA and NHA; the main reason might be that the three materials increased soil pH, reduced exchangeable acid, and exchangeable aluminum content and increased the fixation capacity of soil to heavy metals [16]. The results showed that there was a significant negative correlation between soil pH and the EXC fraction of Cu and Cd, indicating that the soil pH played an important role in affecting the activity of heavy metals in soil. In addition, hydroxyapatite could reduce the activity of heavy metals mainly through ion exchange, surface complexation, and coprecipitation [39]. More importantly, as a phosphorus-containing material, hydroxyapatite can reduce the availability of Cu and Cd in soil by forming phosphate precipitation [40]. Meanwhile, there are differences in the mechanism of adsorption and fixation of Cu and Cd by hydroxyapatite with different particle sizes; the surface and structural characteristics of MHA and NHA make it have more adsorption sites and improve the adsorption capacity of Cu and Cd [14]. Generally, the smaller the particle size, the larger the specific surface area and surface energy and the stronger adsorption and fixation ability to heavy metals [13]. However, there was no significant difference of activity reduce for Cu and Cd between MHA and NHA in our study.

The exchangeable fraction (EXC) is a suitable parameter to evaluate the bioavailability and environmental toxicity of heavy metals [41]. In this study, the exchangeable fraction (EXC) of Cu and Cd was significantly decreased, while the Fe-Mn oxides-bound and CA fraction of Cu and Cd were significantly increased after the application of these three amendments. The results indicated that all these three different particle sizes of hydroxyapatite could significantly decrease the bioavailability of Cu and Cd in this contaminated soil.

### 3.3. Distribution of Cu and Cd in Aggregate Fractions

Soil aggregate is made up of individual soil particles and organic matter whose size and stability can exert direct effects on soil's physical, chemical, and biological characteristics and plant growth [42]. The composition of soil aggregates is listed in Table 4. For soil mechanical-stable aggregates, the application of the three kinds of amendments mainly increased the 1-2 mm aggregate (28.9%–57.2%) and reduced the <0.25 mm aggregate (2.62%–15.1%). For soil water-stable aggregates, the combined remediation mainly increased the >2 mm aggregate (31.5%–47.0%) and reduced the 0.053–0.25 mm aggregate (9.48%–27.2%). This study showed that the content of aggregates sized >2 mm was greatly increased after the remediation, and the increase of larger aggregate content was beneficial to improving the mechanical stability and water stability of soil. The stability of the soil aggregates was closely related to the soil organic carbon, which could promote the cementation of soil particles [43]. In this study, the application of these three amendments promoted the vegetation restoration which increased the amount of litter and root exudates, thus benefiting the accumulation of organic carbon (Table 1), and consequently improved the content of stability aggregates [44].

This study was mainly focused on examining the heavy metal in the wet soil aggregate fractions, which have been shown reliable to study changes in the distribution of heavy metals in long-term soil use [45]. Both maximum Cu and Cd concentration occurred in <0.053 mm aggregate, followed by the 0.25–2 mm, >2 mm, and 0.053–0.25 mm aggregate (Table 5). The results showed that the application of these three hydroxyapatites could increase the concentration of Cu and Cd in all particle size aggregates, and this change reached significant level in 0.25–2 mm (37.2%–63.5%) aggregate for Cu and in 0.25–2 mm (27.5%–104%) and <0.053 mm (26.2%–87.6%) aggregate for Cd.

The highest concentrations of heavy metals were found in the smallest aggregates (<0.053 mm), probably due to the larger surface area of the small aggregates [46]. The silt and clay were the main components in the <0.053 mm sized fraction, where metals might act as the binding agents for the clay-polyvalent metal-organic matter complexes [47]. Thus, heavy metals could easily accumulate on their large surfaces by adsorption, forming chelating complexes with the organic mineral colloidal particles in the finest fractions [48]. Furthermore, the Cu and Cd concentrations in all the wet soil aggregate fractions of the treatments were slightly increased, which might be attributed to the higher content of total Cu and Cd in the treated whole soil than CK (Table 1).

In addition, although the concentration of Cu and Cd in the <0.053 mm sized aggregates was the fundamental part, the mass loading levels were not predominant (Figure 2), and the 0.25–2 mm, 0.053–0.25 mm, and >2 mm aggregates played important roles as Cu and Cd reservoirs in aggregate. This was due partly to the higher aggregate content of the 0.25–2 mm, 0.053–0.25 mm, and >2 mm aggregates. Meanwhile, the content of heavy metals in the atmospheric deposition was high in this area, with some of the new input of heavy metals being first adsorbed on the surface of the microaggregates and then the fine soil particles, leading to a high concentration of heavy metals and the formation of macroaggregates under the action of SOC [49]. In our remediation, the content of SOC was increased because of the growth of plants, which subsequently promoted the transition of soil from the microaggregates to macroaggregates, eventually leading to the transfer of heavy metals from microaggregates into macroaggregates. This might be the possible reason for the increased mass loading levels of Cu and Cd in the >0.053 mm sized aggregates following the chemical-plant treatments. This process made the load capacity of heavy metals in larger aggregates increase gradually, while the mobility of heavy metals in larger aggregates was relatively weak [50], which reduced the migration ability of heavy metals in the environment. As a result, the accumulation of Cu and Cd in aggregates after application of amendments increased the total amount of heavy metals in soil due to the input of heavy metals in this area. Therefore, although the passivation remediation could reduce the mobility and biological activity of heavy metals in areas where pollution sources still existed, there was a risk of increasing the total amount of heavy metals in the soil.

### 3.4. Colloids and Cu and Cd in Colloids

The content of soil colloid was significantly increased by all the three particle size hydroxyapatite (Table 6), and the order of increase was MHA (130%) > NHA (124%) > HA (61.8%). The results illustrated that the addition of hydroxyapatite might affect the composition of soil particles and lead to the transformation between soil particles. Although the hydroxyapatite had similar chemical composition, there were big differences in their particle sizes. Due to the small particle size of microhydroxyapatite and nanohydroxyapatite, they might become a part of soil colloid after adding into soil, which might lead to the content of soil colloid in MHA and NHA treatment higher than that in HA treatment. However, because of the small size, large specific surface area, and the lack of adjacent coordination atoms on the surface, nanohydroxyapatite had high activity, which leads to the aggregation of nanohydroxyapatite [51]. Therefore, the colloid content of NHA treatment was slightly lower than that of MHA treatment.

Hydroxyapatite with three different particle sizes could significantly reduce the concentration of Cu in colloid, and the order of reduction is MHA (20.3%) > NHA (15.2%) > HA (14.2%) (Table 6). The concentration of Cd in soil colloid was significantly reduced by the addition of hydroxyapatite (22.5%), but MHA and NHA had no significant effect on the Cd concentration in soil colloid. The addition of amendments could reduce the concentration of Cu and Cd in the colloid, which might be due to the transformation of other particle size soils into smaller soil colloids. While the contents of Cu and Cd in larger particle size soils were lower, this transformation reduced the concentrations of Cu and Cd in soil colloids. More importantly, we found that the concentration of Cu and Cd in colloid was much higher than that in whole soil (Tables 1 and 6), and the concentration of Cu and Cd in colloid was 3.05–3.81 and 3.99–5.68 times higher than that in whole soil. This was similar to Ajmone-Marsan who found that Cr, Cu, Ni, Pb, and Zn in the soils of five European cities were mainly concentrated in soil particles less than 10 *μ*m [52]. This might be due to the larger specific surface area and more active sites in soil colloids, which lead to the enhancement of adsorption capacity of soil colloids for heavy metals [43].

The product of soil colloid content and heavy metal concentration in colloid is regarded as the fixed component of soil colloid heavy metal, and its ratio to total heavy metal in soil is regarded as the colloidal heavy metal distribution percentage. All of three particle size hydroxyapatite could significantly increase the colloidal Cu and Cd distribution percentage, and the increase range was 49.9%–120% and 30.3%–181%, respectively (Figure 3). These results indicated that 3 kinds of hydroxyapatite lead more heavy metals to soil colloid, and the change of soil colloid content caused by hydroxyapatite might be the main reason for the different colloidal Cu and Cd distribution percentage. Particulate water and air transport are important ways of heavy metal migration in soil environment [53], which are closely related to water transport and workers' physical contact, respectively [54]. The increase of colloidal Cu and Cd distribution percentage could greatly improve the colloid migration and dust migration possibility of heavy metal. Although many studies have shown that different particle sizes of hydroxyapatite have great passivation effect on heavy metals [55, 56], these results indicated that different particle sizes of hydroxyapatite can reduce the risk of heavy metals to organisms, but the possibility of heavy metals migration with soil colloids has not been considered. Therefore, it is necessary to pay attention to soil colloid content and colloidal heavy metal distribution percentage during soil remediation.

## 4. Conclusion

Heavy metal was distributed and migrated as an important component of the contaminated soil ecosystem, whose composition and fraction changed significantly in response to a one-time application of HA, MHA, and NHA combined with the planting of *Elsholtzia splendens* in the smelter-impacted soil. The application of three different particle sizes of hydroxyapatite significantly raised the soil pH, total phosphorus, and SOC. The addition of HA, MHA, and NHA could reduce the EXC fraction of Cu and Cd in soil, thus reducing the bioavailability of heavy metals in soil. In addition, the concentration of Cu and Cd in aggregates was significantly increased, which might cause the increasing of the total Cu and Cd in the soil where the pollution sources still existed. What is more, the content of soil colloid and the colloidal Cu and Cd distribution percentage had been significantly increased after 4 years of one-time addition of three different particle sizes of hydroxyapatite, which might greatly increase the colloid migration and dust migration possibility of Cu and Cd. Therefore, it is not only necessary to focus on the biological activity of heavy metals but also needed to pay attention to monitoring of soil colloid content and colloidal heavy metal distribution percentage, distribution of heavy metals in aggregates, and other indicators related to the distribution and migration of heavy metals, especially in areas where pollution sources still exist.

## Figures and Tables

**Figure 1:** The (a) ordinary particle size of hydroxyapatite (HA) and TEM imaging of (b) microhydroxyapatite (MAP) and (c) nanohydroxyapatite (NAP).

**Figure 2:** Cu and Cd mass loading values in soil aggregates (%).

**Figure 3:** Cu and Cd distribution ratios in soil colloid.

**Table 1:** Soil chemical properties and the biomass of *Elsholtzia splendens* under different treatments.

Treatment	CK	HA	MHA	NHA
Soil pH^a^	4.80 ± 0.075b^b^	5.97 ± 0.070a	5.93 ± 0.074a	5.98 ± 0.133a
TCu (mg kg^−1^ soil)^a^	517 ± 11.9a	487 ± 32.3a	514 ± 11.1a	512 ± 69.9a
TCd (*μ*g kg^−1^ soil)^a^	409 ± 3.64a	413 ± 8.46a	427 ± 18.9a	419 ± 9.67a
TN (g kg^−1^ soil)^a^	1.34 ± 0.134a	1.37 ± 0.218a	1.44 ± 0.045a	1.42 ± 0.023a
TP (g kg^−1^ soil)^a^	0.263 ± 0.0322c	0.400 ± 0.0264b	0.340 ± 0.0557bc	0.527 ± 0.0322a
TK (g kg^−1^ soil)^a^	2.38 ± 0.362a	2.42 ± 0.0472a	2.60 ± 0.214a	2.46 ± 0.129a
AN (mg kg^−1^ soil)^a^	33.6 ± 2.11c	45.5 ± 2.36 b	55.2 ± 1.71a	48.9 ± 1.58 b
AP (mg kg^−1^ soil)^a^	93.4 ± 6.11d	152 ± 13.6c	298 ± 16.6 b	359 ± 7.66a
AK (mg kg^−1^ soil)^a^	60.9 ± 10.7b	84.7 ± 6.33a	71.8 ± 6.14ab	66.7 ± 3.33ab
SOC (g kg^−1^ soil)^a^	16.5 ± 0.417b	18.6 ± 0.540a	18.3 ± 0.432a	19.2 ± 0.975a
Plant (kg plot^−1^)^a^	NG^c^	7.20 ± 0.291a	7.24 ± 0.555a	8.07 ± 0.929a

^a^TCu: total copper; TCd: total cadmium; TN: total nitrogen; TP: total phosphorus; TK: total potassium; AN: available nitrogen; AP: available phosphorus; AK: available potassium; SOC: soil organic carbon; plant: the biomass of *Elsholtzia splendens*. ^b^Different letters indicate significant difference between treatments detected by Tukey's multiple test (*p* < 0.05). ^c^NG indicates the tested plants did not grow under this treatment.

**Table 2:** Effects of apatite, microhydroxyapatite, and nanohydroxyapatite application on Cu fractions.

Cu (mg kg^−1^)	EXC^a^	CA	Fe-Mn	OM	RES	Total
CK	115 ± 16.5a^b^	47.2 ± 4.64 b	93.9 ± 6.09 b	97.9 ± 7.69a	147 ± 9.07a	517 ± 11.9a
HA	38.5 ± 10.1bc	88.5 ± 16.3a	143 ± 31.3ab	94.7 ± 15.3a	126 ± 21.6a	487 ± 32.3a
MHA	30.2 ± 4.71c	101 ± 5.88a	161 ± 4.52a	109 ± 7.69a	125 ± 8.70a	514 ± 11.1a
NHA	22.9 ± 9.14c	91.6 ± 25.5a	148 ± 33.1ab	100 ± 15.8a	161 ± 28.9a	512 ± 69.9a

^a^EXC: exchangeable fraction; CA: carbonate-bound fraction; Fe-Mn: Fe-Mn oxides-bound fraction; OM: organic matter-bound fraction; RES: residual fraction. ^b^Different letters indicate significant difference between treatments detected by Tukey's multiple test (*p* < 0.05).

**Table 3:** Effects of apatite, microhydroxyapatite, and nanohydroxyapatite application on Cd fractions.

Cd (*μ*g kg^−1^)	EXC	CA	Fe-Mn	OM	RES	Total
CK	159 ± 29.4a	14.9 ± 3.85b	30.2 ± 8.09b	38.8 ± 15.3a	162 ± 46.5a	409 ± 3.64a
HA	126 ± 6.75ab	17.0 ± 5.46b	53.8 ± 1.37a	32.7 ± 10.5a	200 ± 23.2a	413 ± 8.46a
MHA	103 ± 6.77b	21.9 ± 7.81ab	64.7 ± 7.25a	30.0 ± 8.75a	215 ± 23.6a	427 ± 18.9a
NHA	112 ± 13.6b	34.6 ± 3.48a	68.5 ± 10.4a	30.1 ± 3.44a	180 ± 27.0a	419 ± 9.67a

^a^EXC: exchangeable fraction; CA: carbonate-bound fraction; Fe-Mn: Fe-Mn oxides-bound fraction; OM: organic matter-bound fraction; RES: residual fraction. ^b^Different letters indicate significant difference between treatments detected by Tukey's multiple test (*p* < 0.05).

**Table 4:** Composition of aggregates in the soil after the remediation (%).

Treatment	Sizes of the soil mechanical-stable aggregates (%)					
	>5 mm	2–5 mm	1-2 mm	0.5–1 mm	0.25–0.5 mm	<0.25 mm

CK	7.06 ± 1.77a^a^	8.66 ± 1.62a	4.91 ± 1.44b	7.78 ± 0.499a	18.1 ± .870bc	53.5 ± 2.37a
HA	7.54 ± 0.864a	9.59 ± .457a	6.33 ± 0.706ab	6.79 ± 0.854a	17.6 ± .630c	52.1 ± .450ab
MHA	7.39 ± 0.338a	10.6 ± 2.12a	7.72 ± 0.855a	6.87 ± 1.023a	19.8 ± .698ab	47.6 ± 3.85ab
NHA	7.61 ± 1.500a	11.9 ± 2.80a	7.16 ± 0.380ab	7.24 ± 0.940a	20.6 ± .993a	45.4 ± 3.38b

Treatment	Sizes of the soil water-stable aggregates (%)					
	>2 mm		0.25–2 mm		0.053–0.25 mm	<0.053 mm

CK	18.1 ± 0.240b		31.7 ± 2.60ab		46.4 ± 2.23a	3.81 ± 0.165a
HA	23.9 ± 2.33a		29.8 ± 0.781b		42.0 ± 2.23ab	4.25 ± 0.851a
MHA	23.8 ± 0.494a		31.2 ± 0.804b		40.5 ± 0.882b	4.56 ± 0.480a
NHA	26.6 ± 1.02a		35.5 ± 1.29a		33.8 ± 0.812c	4.08 ± 0.544a

^a^Different letters indicate significant difference between treatments detected by Tukey's multiple test (*p* < 0.05).

**Table 5:** Concentrations of Cu and Cd in different size aggregates of wet soil aggregates for different treatments.

Treatment	>2 mm	0.25–2 mm	0.053–0.25 mm	<0.053 mm
	Cu (mg kg^−1^)			
CK	3.73 × 10^2^ ± 44.8a^a^	4.38 × 10^2^ ± 37.5b	2.41 × 10^2^ ± 3.02a	5.77 × 10^2^ ± 23.4a
HA	4.96 × 10^2^ ± 89.4a	7.16 × 10^2^ ± 49.8a	3.24 × 10^2^ ± 55.2a	7.38 × 10^2^ ± 58.3a
MHA	4.67 × 10^2^ ± 12.5a	6.01 × 10^2^ ± 55.5b	3.27 × 10^2^ ± 8.96a	6.98 × 10^2^ ± 96.1a
NHA	4.19 × 10^2^ ± 64.8a	6.06 × 10^2^ ± 62.8b	2.99 × 10^2^ ± 60.8a	6.32 × 10^2^ ± 67.4a

	Cd (*μ*g kg^−1^)			
CK	2.87 × 10^2^ ± 16.4a	2.91 × 10^2^ ± 47.8b	2.21 × 10^2^ ± 43.5a	4.93 × 10^2^ ± 16.8b
HA	4.12 × 10^2^ ± 83.8a	5.49 × 10^2^ ± 123ab	3.45 × 10^2^ ± 43.2a	9.25 × 10^2^ ± 18.6a
MHA	3.42 × 10^2^ ± 28.4a	5.94 × 10^2^ ± 83.7a	3.36 × 10^2^ ± 8.29a	6.22 × 10^2^ ± 261ab
NHA	3.41 × 10^2^ ± 82.1a	3.71 × 10^2^ ± 136ab	3.10 × 10^2^ ± 86.3a	6.45 × 10^2^ ± 176ab

^a^Different letters indicate significant difference between treatments detected by Tukey's multiple test (*p* < 0.05).

**Table 6:** Soil colloid content and Cu/Cd concentration in soil colloid.

Treatment	Colloid content (g kg^−1^)	Cu concentration in colloid (mg·kg^−1^)	Cd concentration in colloid (*μ*g·kg^−1^)
CK	51.3 ± 5.90c	1.97 × 10^3^ ± 270a	2.13 × 10^3^ ± 289a
HA	83.0 ± 4.50b	1.69 × 10^3^ ± 118b	1.65 × 10^3^ ± 101b
MHA	118 ± 9.45a	1.57 × 10^3^ ± 141c	2.33 × 10^3^ ± 189a
NHA	115 ± 3.60a	1.67 × 10^3^ ± 74.6b	2.38 × 10^3^ ± 91.9a

## Data Availability

All the data used to support the findings of this study are available from the corresponding author upon request.

## References

[1] Sun Y., Li H., Guo G., Semple K. T., Jones K. C. (2019). Soil contamination in China: current priorities, defining background levels and standards for heavy metals. *Journal of Environmental Management*.

[2] Zhuo H., Fu S., Liu H., Song H., Ren L. (2019). Soil heavy metal contamination and health risk assessment associated with development zones in Shandong, China. *Environmental Science and Pollution Research*.

[3] Obiora S. C., Chukwu A., Davies T. C. (2016). Heavy metals and health risk assessment of arable soils and food crops around Pb–Zn mining localities in Enyigba, Southeastern Nigeria. *Journal of African Earth Sciences*.

[4] Meng J., Tao M., Wang L., Liu X., Xu J. (2018). Changes in heavy metal bioavailability and speciation from a Pb-Zn mining soil amended with biochars from co-pyrolysis of rice straw and swine manure. *The Science of the Total Environment*.

[5] Lwin C. S., Seo B.-H., Kim H.-U., Owens G., Kim K.-R. (2018). Application of soil amendments to contaminated soils for heavy metal immobilization and improved soil quality-a critical review. *Soil Science & Plant Nutrition*.

[6] Li B., Yang L., Wang C. Q., Zheng S. Q., Xiao R., Guo Y. (2019). Effects of organic-inorganic amendments on the cadmium fraction in soil and its accumulation in rice (*Oryza sativa L*.). *Environmental Science and Pollution Research*.

[7] Valipour M., Shahbazi K., Khanmirzaei A. (2016). Chemical immobilization of lead, cadmium, copper, and nickel in contaminated soils by phosphate amendments. *Clean-Soil, Air, Water*.

[8] Guo F., Ding C., Zhou Z., Huang G., Wang X. (2018). Stability of immobilization remediation of several amendments on cadmium contaminated soils as affected by simulated soil acidification. *Ecotoxicology and Environmental Safety*.

[9] Xu L., Xing X., Liang J., Peng J., Zhou J. (2019). In situ phytoremediation of copper and cadmium in a co-contaminated soil and its biological and physical effects. *RSC Advances*.

[10] Komárek M., Vaněk A., Ettler V. (2013). Chemical stabilization of metals and arsenic in contaminated soils using oxides-a review. *Environmental Pollution*.

[11] Cui H., Zhang W., Zhou J. (2018). Availability and vertical distribution of Cu, Cd, Ca, and P in soil as influenced by lime and apatite with different dosages: a 7-year field study. *Environmental Science and Pollution Research*.

[12] Xing J., Hu T., Cang L., Zhou D. (2016). Remediation of copper contaminated soil by using different particle sizes of apatite: a field experiment. *SpringerPlus*.

[13] Chen S. B., Zhu Y. G., Ma Y. B. (2006). The effect of grain size of rock phosphate amendment on metal immobilization in contaminated soils. *Journal of Hazardous Materials*.

[14] Dong A., Ye X., Li H., Zhang Y., Wang G. (2016). Micro/nanostructured hydroxyapatite structurally enhances the immobilization for Cu and Cd in contaminated soil. *Journal of Soils and Sediments*.

[15] Zhang Z., Li M., Chen W., Zhu S., Liu N., Zhu L. (2010). Immobilization of lead and cadmium from aqueous solution and contaminated sediment using nano-hydroxyapatite. *Environmental Pollution*.

[16] Cui H., Shi Y., Zhou J., Chu H., Cang L., Zhou D. (2018). Effect of different grain sizes of hydroxyapatite on soil heavy metal bioavailability and microbial community composition. *Agriculture, Ecosystems & Environment*.

[17] Cui H., Zhou J., Zhao Q. (2013). Fractions of Cu, Cd, and enzyme activities in a contaminated soil as affected by applications of micro-and nanohydroxyapatite. *Journal of Soils and Sediments*.

[18] Walkley A., Black I. A. (1934). An examination of the degtjareff method for determining soil organic matter, and a proposed modification of the chromic acid titration method. *Soil Science*.

[19] Page A. L., Miller R. H., Keeney D. R. (1982). *Methods of Soil Analysis: Chemical and Microbiological Properties*.

[20] Olsen S. R. (1954). *Estimation of Available Phosphorus in Soils by Extraction with Sodium Bicarbonate*.

[21] Hinesly T. D., Redborg K. E., Ziegler E. L., Alexander J. D. (1982). Effect of soil cation exchange capacity on the uptake of cadmium by corn. *Soil Science Society of America Journal*.

[22] Elliott E. T. (1986). Aggregate structure and carbon, nitrogen, and phosphorus in native and cultivated soils. *Soil Science Society of America Journal*.

[23] Panettieri M., Berns A. E., Knicker H., Murillo J. M., Madejón E. (2015). Evaluation of seasonal variability of soil biogeochemical properties in aggregate-size fractioned soil under different tillages. *Soil and Tillage Research*.

[24] Gijsman A. (1996). Soil aggregate stability and soil organic matter fractions under agropastoral systems established in native savanna. *Soil Research*.

[25] Xu L., Cui H., Zheng X. (2017). Changes in the heavy metal distributions in whole soil and aggregates affected by the application of alkaline materials and phytoremediation. *RSC Advances*.

[26] Tessier A., Campbell P. G. C., Bisson M. (1979). Sequential extraction procedure for the speciation of particulate trace metals. *Analytical Chemistry*.

[27] Klitzke S., Lang F. (2007). Hydrophobicity of soil colloids and heavy metal mobilization. *Journal of Environmental Quality*.

[28] Hu J. D., Ya-Ting S., Xue-Jun W. (2009). Release and mobilization of soil colloid in the natural soil packed column with various water saturations. *Journal of Agro-Environment Science*.

[29] Wei L., Wang S., Zuo Q., Liang S., Shen S., Zhao C. (2016). Nano-hydroxyapatite alleviates the detrimental effects of heavy metals on plant growth and soil microbes in e-waste-contaminated soil. *Environmental Sciences: Processes & Impacts*.

[30] Mwafulirwa L., Baggs E. M., Morley N., Paterson E. (2019). Ryegrass root and shoot residues differentially affect short-term priming of soil organic matter and net soil C-balance. *European Journal of Soil Biology*.

[31] Zhu Z., Ge T., Xiao M. (2017). Belowground carbon allocation and dynamics under rice cultivation depends on soil organic matter content. *Plant and Soil*.

[32] Tao M. J., Zhou J., Liang J. N., Cui H. B., Xu L. (2014). Study on atmospheric deposition characteristics of Cu and Cd in summer around one smelting factory. *Environmental Monitoring in China*.

[33] Cui H., Fan Y., Xu L. (2016). Sustainability of in situ remediation of Cu-and Cd-contaminated soils with one-time application of amendments in Guixi, China. *Journal of Soils and Sediments*.

[34] Cui H., Zhou J., Si Y. (2014). Immobilization of Cu and Cd in a contaminated soil: one-and four-year field effects. *Journal of Soils and Sediments*.

[35] Puga A. P., Azevedo Melo L. C., De Abreu C. A., Coscione A. R., Paz-Ferreiro J. (2016). Leaching and fractionation of heavy metals in mining soils amended with biochar. *Soil and Tillage Research*.

[36] He L., Zhong H., Liu G., Dai Z., Brookes P. C., Xu J. (2019). Remediation of heavy metal contaminated soils by biochar: mechanisms, potential risks and applications in China. *Environmental Pollution*.

[37] Cao X., Ma L. Q., Rhue D. R., Appel C. S. (2004). Mechanisms of lead, copper, and zinc retention by phosphate rock. *Environmental Pollution*.

[38] Siebers N., Kruse J., Leinweber P. (2013). Speciation of phosphorus and cadmium in a contaminated soil amended with bone char: sequential fractionations and XANES spectroscopy. *Water, Air, and Soil Pollution*.

[39] Ferri M., Campisi S., Scavini M., Evangelisti C., Carniti P., Gervasini A. (2018). In-depth study of the mechanism of heavy metal trapping on the surface of hydroxyapatite. *Applied Surface Science*.

[40] Yuan S. D., Li X. Y., Ye M. (2017). Research on the rapid preparation process of nano hydroxyapatite powder by chemical precipitation. *Journal of Jiamusi University*.

[41] Zhang H., Ma G., Sun L., Li H. (2017). Effect of alkaline material on phytotoxicity and bioavailability of Cu, Cd, Pb and Zn in stabilized sewage sludge. *Environmental Technology*.

[42] Vezzani F. M., Anderson C., Meenken E., Gillespie R., Peterson M., Beare M. H. (2018). The importance of plants to development and maintenance of soil structure, microbial communities and ecosystem functions. *Soil and Tillage Research*.

[43] Zhao J., Chen S., Hu R., Li Y. (2017). Aggregate stability and size distribution of red soils under different land uses integrally regulated by soil organic matter, and iron and aluminum oxides. *Soil and Tillage Research*.

[44] Adesodun J. K., Nuga B. O., Udom B. E. (2016). Water-stable aggregates and aggregate-associated organic carbon and nitrogen after three annual applications of poultry manure and spent mushroom wastes. *Applied Soil Ecology*.

[45] Hardie M., Clothier B., Bound S., Oliver G., Close D. (2014). Does biochar influence soil physical properties and soil water availability?. *Plant and Soil*.

[46] Xiao R., Zhang M. X., Yao X., Ma Z. W., Yu F. H., Bai J. (2016). Heavy metal distribution in different soil aggregate size classes from restored brackish marsh, oil exploitation zone, and tidal mud flat of the Yellow River Delta. *Journal of Soils and Sediments*.

[47] Shen L. C., Lo A., Nguyen X. T., Hankins N. P. (2016). Recovery of heavy metal ions and recycle of removal agent in the polymer-surfactant aggregate process. *Separation and Purification Technology*.

[48] Li H., Han X., Wang F., Qiao Y., Xing B. (2007). Impact of soil management on organic carbon content and aggregate stability. *Communications in Soil Science and Plant Analysis*.

[49] Sutherland R. A. (2003). Lead in grain size fractions of road-deposited sediment. *Environmental Pollution*.

[50] Yin Y. M., Zhao W. T., Huang T., Cheng S. G., Zhao Z. L., Cong-Cong Y. U. (2018). Distribution characteristics and health risk assessment of heavy metals in a soil-rice system in an E-waste dismantling area. *Environmental Ence*.

[51] Gilbert B., Ono R. K., Ching K. A., Kim C. S. (2009). The effects of nanoparticle aggregation processes on aggregate structure and metal uptake. *Journal of Colloid and Interface Science*.

[52] Ajmone-Marsan F., Biasioli M., Kralj T. (2008). Metals in particle-size fractions of the soils of five European cities. *Environmental Pollution*.

[53] Baumann T., Fruhstorfer P., Klein T., Niessner R. (2006). Colloid and heavy metal transport at landfill sites in direct contact with groundwater. *Water Research*.

[54] Chen G., Zeng G., Du C. (2010). Transfer of heavy metals from compost to red soil and groundwater under simulated rainfall conditions. *Journal of Hazardous Materials*.

[55] Liu H. Y., Zhang Y., Chen N. (2018). Effect of surface characteristics of hydroxyapatite on the remediation passivation effect of heavy metal contaminated soil. *Environmental Chemistry*.

[56] Zhu F., He S., Shang Z. (2019). Effect of vegetables and nano-particle hydroxyapatite on the remediation of cadmium and phosphatase activity in rhizosphere soil through immobilization. *International Journal of Phytoremediation*.

